The article "Taxonomy of Adaptive Neuro-Fuzzy Inference System in Modern Engineering Sciences" was retracted in 2023. Reasons: signs of a paper mill; compromised peer review; unreliable results or conclusions.

# Taxonomy of Adaptive Neuro-Fuzzy Inference System in Modern Engineering Sciences

**DOI:** 10.1155/2021/6455592

**Published:** 2021-09-03

**Authors:** Shivali Chopra, Gaurav Dhiman, Ashutosh Sharma, Mohammad Shabaz, Pratyush Shukla, Mohit Arora

**Affiliations:** ^1^Lovely Professional University, Phagwara, Punjab, India; ^2^Government Bikram College of Commerce, Patiala, Punjab, India; ^3^Institute of Computer Technology and Information, Security Southern Federal University, Taganrog, Russia; ^4^Arba Minch University, Arba Minch, Ethiopia; ^5^Institute of Engineering and Technology, Chitkara University, Punjab, Chandigarh, India; ^6^New York University, New York City, NY, USA

## Abstract

Adaptive Neuro-Fuzzy Inference System (ANFIS) blends advantages of both Artificial Neural Networks (ANNs) and Fuzzy Logic (FL) in a single framework. It provides accelerated learning capacity and adaptive interpretation capabilities to model complex patterns and apprehends nonlinear relationships. ANFIS has been applied and practiced in various domains and provided solutions to commonly recurring problems with improved time and space complexity. Standard ANFIS has certain limitations such as high computational expense, loss of interpretability in larger inputs, curse of dimensionality, and selection of appropriate membership functions. This paper summarizes that the standard ANFIS is unsuitable for complex human tasks that require precise handling of machines and systems. The state-of-the-art and practice research questions have been discussed, which primarily focus on the applicability of ANFIS in the diversifying field of engineering sciences. We conclude that the standard ANFIS architecture is vastly improved when amalgamated with metaheuristic techniques and further moderated with nature-inspired algorithms through calibration and tuning of parameters. It is significant in adapting and automating complex engineering tasks that currently depend on human discretion, prominent in the mechanical, electrical, and geological fields.

## 1. Introduction

The machine learning domain contains a wide variety of models based on the learning ability, adaptiveness, complexity, and scalability. Some of the popular techniques are Fuzzy Logic, Extreme Learning Machine, Boosting, Bagging, Artificial Neural Networks, etc. Many researchers used machine learning algorithms based on these techniques like regression, decision trees, random forest, stochastic gradient, Support Vector Regressors (SVR), etc. and its ensembles other optimization techniques [1]. Hybrids of such techniques have been proposed and developed that tend to solve their deficiencies as well as provide robustness and powerful prediction capabilities. One such technique with the inherent potential of both neural networks and fuzzy systems is ANFIS [2], which provides great estimation accuracy, i.e., low Mean Magnitude of Relative Error (MMRE) and high Prediction (PRED).

The article "Taxonomy of Adaptive Neuro-Fuzzy Inference System in Modern Engineering Sciences" was retracted in 2023. Reasons: signs of a paper mill; compromised peer review; unreliable results or conclusions.

ANFIS is the most popular neuro-fuzzy model for approximating highly complex, nonlinear systems. The key aspects of ANFIS are the accuracy using the precise fuzzy modelling and interpretability, which improves its generalization ability. ANFIS has gained prominence amongst researchers for its robustness in modelling fuzzy sets into crisp inputs and providing crisp outputs from the fuzzy rules for reasoning purpose. Ironically, ANFIS has to balance the accuracy-interpretability trade-off [3]. The advantages and disadvantages of ANFIS have been discussed in Table 1. It is of considerable importance in ANFIS to find the type and number of membership functions, suitable to the process or system. ANFIS is generally very efficient until the number of inputs is below five [4]. Modern engineering systems have more inputs as the complexity of the problem increases, for instance, signal processing in a highly chaotic environment, flood susceptibility detection in watershed management, precise coordination of I&C systems in a nuclear plant, etc.

Originally, ANFIS was designed with the use of Gradient Descent (GD) and Least Square Estimation (LSE) for optimizing its parameters. GD is a very popular optimization algorithm that is commonly used to train neural networks. It uses backpropagation method to calculate gradients, thus having the easiest system of computation. LSE method of optimization is very common in regression-based models. It calculates the least sum of squared errors, finding the optimal coefficients of the errors. However, these are not efficient to model complex engineering tasks that are highly nonlinear in nature and require precise control over the systems. Then, it provides an opportunity to improve the capability of ANFIS.

GD is a basic optimization algorithm that suffers when the nonlinearity of the system increases. Hence, it may fail to find the global optima and remain trapped at local minima. For large datasets, redundant computations are performed for the same set of training data, slowing the convergence. It has high computational cost, when frequently updating the weights of the neural network, wasting computational resources.

LSE is a rudimentary optimization method that is very sensitive to outliers. Its performance is affected when the data is not normally distributed, which leads to overfitting in most cases. Also, LSE is more computationally expensive than GD, becoming slower with increasing complexity of the system.

The article "Taxonomy of Adaptive Neuro-Fuzzy Inference System in Modern Engineering Sciences" was retracted in 2023. Reasons: signs of a paper mill; compromised peer review; unreliable results or conclusions.

ANFIS is plagued by issues inherent in its fundamental structure. The optimization algorithms thus used are instrumental in altering the performance of ANFIS. Metaheuristic techniques assist ANFIS in searching for solutions for optimal and accurate predictions. Metaheuristic techniques provide a high-level and problem-independent set of directives to develop optimization techniques. These techniques have been found superior to the traditional techniques of optimization. Their goal is to compute a “good enough” solution in a “small enough” computing time not subjected to combinatorial explosion [5]. Hence, the solution obtained is quick and efficient, enabling optimization of the problem definition at hand. The various research papers that have been reviewed have hybridized the standard ANFIS architecture to include such metaheuristic algorithms for optimizing ANFIS premise and consequent parameters [6]. These optimization techniques can improve the standard ANFIS architecture [7, 8].

This paper has been divided into 4 sections: Section 1 provides Introduction, Section 2 contains the review methodology, Section 3 contains the Results and Discussions, and Section 4 describes the Conclusion and Future research directions.

This table presents the advantages and disadvantages of the original ANFIS system, as designed by J.S. Roger Jang. These limitations are unsuitable for use in modern, real-world systems and, hence, need to be resolved to be deployed in production on the machines.

## 2. Method

In this section, we have discussed the classic ANFIS [2], various research questions, review *inclusion* and *exclusion* criteria, data sources description, and study selection process [9]. The steps are shown in Figure 1.

### 2.1. Adaptive Neuro-Fuzzy Inference System

Adaptive Neuro-Fuzzy Inference Systems, developed in 1993 by J.S. Roger Jang, are widely regarded as a universal estimator or Takagi-Sugeno Fuzzy System. The Takagi-Sugeno Fuzzy model is a Type 3 Fuzzy Inference System, where the rule outputs are a linear combination of input variable along with a constant, and the final output is the weighted average of every rule's output.

The IF-THEN rules for a 3-input Takagi-Sugeno system are described as follows.

- Rule 1: IF *x* is *A*_1_, *y* is *B*_1_, *z* is *C*_1_, THEN *f*_1_=*p*_1_*x*+*q*_1_*y*+*r*_1_*z*+*s*_1_
- Rule 2: IF *x* is *A*_2_, *y* is *B*_2_, *z* is *C*_2_, THEN *f*_2_=*p*_2_*x*+*q*_2_*y*+*r*_2_*z*+*s*_2_
- Rule 3: IF *x* is *A*_3_, *y* is *B*_3_, *z* is *C*_3_, THEN *f*_3_=*p*_3_*x*+*q*_3_*y*+*r*_3_*z*+*s*_3_
- where *x*, y, *z* are the inputs in the crisp set; *A*_*i*_, *B*_*i*_, *C*_*i*_ are the linguistic labels; *p*_*i*_, *q*_*i*_, *r*_*i*_ are the consequent parameters; *f*_1_, *f*_2_, *f*_3_ are the output fuzzy membership functions.

The article "Taxonomy of Adaptive Neuro-Fuzzy Inference System in Modern Engineering Sciences" was retracted in 2023. Reasons: signs of a paper mill; compromised peer review; unreliable results or conclusions.

The standard ANFIS architecture, as given in Figure 2, consists of five layers of interconnected neurons, evident of artificial neural networks having alike functionalities. The architecture is briefly explained as follows.

#### 2.1.1. Layer 1

It is the Fuzzification Layer where each neuron is an adaptive node and holds the fuzzy value of the crisp inputs.

The node output is calculated as follows:

(1) $$\begin{array}{c} O_{i}^{1}=\left\{\begin{array}{cc} \mu_{Ai}\left(x\right), & \forall i=1,2,\\ \mu_{Bi-2}\left(x\right), & \forall i=3,4,\\ \mu_{Ci-4}\left(x\right), & \forall i=5,6, \end{array}\right) \end{array}$$

where *μ* is a membership function for the fuzzy sets *A*_*i*_, *B*_*i*_, *C*_*i*_. Numerous membership functions exist, i.e., Gaussian, Trapezoidal, Triangular, etc. We prefer a bell-shaped function in ANFIS. Hence, the Gaussian function is the optimum choice. The formula for Gaussian function is

(2) $$\begin{array}{c} f\left(x\right)=a\cdot \;\exp\left\{-\frac{{\left(x-b\right)}^{2}}{2c^{2}}\right\}, \end{array}$$

where *a*, *b*, *c* are the premise parameters for the membership functions of ANFIS.

#### 2.1.2. Layer 2

This is an Implication Layer where the neurons contain the product of inputs, i.e., the weight of premise parameters. The node output is calculated as follows:

(3) $$\begin{array}{c} O_{i}^{2}=w_{i}=\mu_{Ai}\left(x\right)\cdot \mu_{Bi}\left(x\right)\cdot \mu_{Ci}\left(x\right),\;\forall i=1,2,3, \end{array}$$

where *w*_*i*_ is the weight of the neuron.

#### 2.1.3. Layer 3

It is Normalizing Layer where the neurons are fixed and are normalized by the sum of weights of all neurons in this layer. The node output is calculated as follows:

(4) $$\begin{array}{c} O_{i}^{3}=\bar{w_{i}}=\frac{w_{i}}{\Sigma w_{i}},\;\forall i=1,2,3, \end{array}$$

where $\bar{w_{i}}$ is the normalized weight of the neuron.

#### 2.1.4. Layer 4

This is the Defuzzification Layer where each neuron is also an adaptive node and holds the consequent parameters of the architecture. The node output is calculated as follows:

(5) $$\begin{array}{c} O_{i}^{4}=\bar{w_{i}}f_{i}=\bar{w_{i}}\cdot \left(p_{i}x+q_{i}y+r_{i}z+s_{i}\right),\;\forall i=1,2,3. \end{array}$$

#### 2.1.5. Layer 5

It is an Output Layer where a single neuron is present for output, which is the sum of all the inputs. The node output is calculated as follows:

(6) $$\begin{array}{c} O_{i}^{5}=f\left(x,y,z\right)=\Sigma_{i}\bar{w_{i}}f_{i}=\frac{\Sigma_{i}w_{i}f_{i}}{\Sigma_{i}w_{i}},\;\forall i=1,2,3. \end{array}$$

Classical ANFIS favors hybrid learning process, where parameters are updated through two passes and use two different optimization algorithms.

The article "Taxonomy of Adaptive Neuro-Fuzzy Inference System in Modern Engineering Sciences" was retracted in 2023. Reasons: signs of a paper mill; compromised peer review; unreliable results or conclusions.

During the forward pass, the consequent parameters are updated, when the inputs are provided to ANFIS, and the premise parameters are kept fixed, using LSE, the consequent parameters are updated in Layer 4, and the final output is calculated accordingly.

As the final output is calculated, the backward pass starts, during which the error is propagated back to Layer 1, and the premise parameters are updated. In this pass, the consequent parameters are kept fixed.

### 2.2. Research Questions

This review paper aims to summarize the current implication status of machine learning models. In this context, the following research questions (RQ) are proposed:

  RQ1: What are the various ANFIS hybrids?
  RQ2: What was the purpose of creating a hybrid ANFIS technique?
  RQ3: What areas of applications have utilized ANFIS hybrids in the real world?
  RQ4: What are the various optimization algorithm hybrids of ANFIS?
  RQ5: What are the possible future research directions in context to ANFIS current literature variants?
  RQ6: What are the current trends in research based on ANFIS techniques?
  RQ7: Which hybrid techniques are the most popular for ANFIS implementations?

### 2.3. Search Strategy

We employ two phases to search and download the studies.

#### 2.3.1. Primary Search

Using the primary search phase, we adopt the following procedure:

- Analyze leading terms within research questions
- Detect alternative terms and spelling for the terms
- Check the keywords in relevant books and journals
- Boolean AND to link leading terms and Boolean OR for alternative terms

#### 2.3.2. Secondary Search

In the secondary search phase, references ignored during the primary search are reviewed. The search string used is, Hybrid AND (ANFIS OR “Neuro-Fuzzy” OR optimization) AND techniques AND (using OR with) AND (“Artificial Bee Colony” OR “Ant Colony Optimization” OR “Bat Algorithm” OR “Bees Algorithm” OR “Biogeography Based Optimization” OR “Cultural Algorithm” OR “Colliding Body Optimization” OR “Cuckoo Optimization Algorithm” OR “Crow Search Algorithm” OR “Cat Search Algorithm” OR “Differential Evolution” OR “Firefly Algorithm” OR “Genetic Algorithm” OR “Grey Wolf Optimizer” OR “Harmony Search” OR “Imperialist Competitive Algorithm” OR “Invasive Weed Optimization” OR “Moth Fly Optimization” OR “Mosquito Host Seeking” OR “Particle Swarm Optimization” OR “Simulated Annealing” OR “Satin Bowerbird Optimizer” OR “Subtractive Clustering” OR “Shuffled Frog-Leaping Algorithm” OR “Social Spider Optimization”).

The search strategy has been further refined using alternative terms and spellings in the search string. Boolean strings enable the discovery of all studies available in the databases, whereas the references present in the selected studies can be benefited from any missing studies. Such considerations, and suggestions, allowed us to employ a search string using Boolean operators OR and AND comprising possible alternatives for the terms. Besides, references of the primary studies served as sources for exploration of possible missing studies. The following sources of literature discovery were used for selecting primary studies:

- PLOS One
- IEEE Xplore
- Springer
- ACM Digital Library
- ScienceDirect
- Elsevier

These revered digital libraries are popular in the research community; hence, we found them suitable to include for compiling our data. The studies we focused on are between 1997 and 2019, with publications in the first quarter of 2020 also included. During the primary search phase, we examined and found 48 relevant studies. Afterward, in the secondary search phase, our discussed criteria allowed the identification of 79 additional relevant studies, missed during the initial searches. Thus, we selected 127 studies specific to our SLR, based on the conducted primary and secondary search phases. The title and abstract of these studies were considered for selection.

The article "Taxonomy of Adaptive Neuro-Fuzzy Inference System in Modern Engineering Sciences" was retracted in 2023. Reasons: signs of a paper mill; compromised peer review; unreliable results or conclusions.

### 2.4. Study Selection

Every study identified based on titles and abstracts during the search strategy was moved through two phases for filtering the studies, such that the desired literature was obtained. The first phase contains inclusion and exclusion criteria for selecting studies of relevance and discarding others for our SLR. In the second phase, further filtering of the selected studies is based on the quality assessment criteria. The inclusion/exclusion criteria specific to our SLR are as follows:

#### 2.4.1. Inclusion Criteria

The following are the inclusion criteria:

- Studies that contain hybrid of ANFIS
- Studies that propose novel optimization techniques
- Studies that contain hybrid of optimization techniques

#### 2.4.2. Exclusion Criteria

The following are the exclusion criteria:

- Studies with little relevance in case of similar content
- Studies containing only Deep Learning techniques or Fuzzy Logic techniques
- Studies published as a thesis

### 2.5. Quality Assessment Criteria

Every study was examined against the quality assessment criteria to validate their plausibility and significance. In particular, after the application of the inclusion/exclusion criteria, we have carefully observed the candidate studies relevant to our purpose. Studies having low quality have been vetoed. We have used the following questions to define the criteria for quality assessment.

  Q1. Are the established aims in the research thoroughly defined?
  Q2. Has the study been cited before?
  Q3. Is the experiment applied against benchmark functions or any application areas?
  Q4. Are the algorithms validated against standard accuracy measures?
  Q5. Are optimization techniques provided with comparative analysis?
  Q6. Are limitations catering to the study analyzed explicitly?
  Q7. How recently the study has been published?
  Q8. Are the journals indexed in SCI or Scopus?

The article "Taxonomy of Adaptive Neuro-Fuzzy Inference System in Modern Engineering Sciences" was retracted in 2023. Reasons: signs of a paper mill; compromised peer review; unreliable results or conclusions.

For assessing the quality of the studies based on these criteria, we provide only three answers with the scores given in (7).

(7) $$\begin{array}{c} \text{score}=\left\{\begin{array}{cc} 1, & \text{if }\forall q\in Q=“\text{Yes}\mathrm{”,}\\ 0.5, & \text{if }\forall q\in Q=“\text{Partly}\mathrm{”,}\\ 0, & \text{if }\forall q\in Q=“\text{No}”. \end{array}\right) \end{array}$$

The quality score for a given study is calculated by taking the mean of the scores against the questions answered and considered for selection as per the threshold in

(8) $$\begin{array}{c} \text{mean of scores}=\left\{\begin{array}{cc} \geq 0.6, & \text{if }“\text{Selected}\mathrm{”,}\\ <0.6, & \text{if }“\text{Not selected}\mathrm{”,} \end{array}\right)\in \left[0,1\right]. \end{array}$$

The quality assessment score for the studies is not based on fuzzy linguistic values because of the relative ease provided by the crisp set in our criteria. As we assess the quality based on the mean of the scores in the range defined in (8), it allows a comfortable examination to us. After several rounds of discussion with regards the quality assessment criteria, all the authors acknowledged the proposed system of scoring. To denote the simplicity of the system, we take an example. Suppose a study receives the subsequent quality assessment scores for the eight questions:

  Q1 (1), Q2 (0.5), Q3 (0.5), Q4 (0.5), Q5 (1), Q6 (1), Q7 (1), and Q8 (1)

The total score is 6.5, and their mean is 0.8. This validates the study for selection as it is above the acceptable threshold defined by our system.

In another example, if the following scores are obtained for a particular study:

  Q1 (0.5), Q2 (0.5), Q3 (1), Q4 (0), Q5 (0), Q6 (0.5), Q7 (0.5), and Q8 (1)

The total score is 4 and their mean is 0.5; hence, this study cannot be included and is filtered. In general, with a minimum total score of 5, the study is suitable for selection in the SLR. The application of these quality assessment criteria excluded 11 studies.

### 2.6. Data Extraction

One issue we recognized when searching the studies for SLR was the use of partial terms. For example, some of the studies contained the term particle swarm and genetic, but not optimization or algorithm. Another issue we recognized was the inclusion of terms in the abstract, but not in the title. As we examined further, we found some studies including the terms for comparative purpose, as opposed to being the focus of the studies. It is worth noting that our research questions are not necessarily answered by all the selected studies. Such note of importance prompted us to analyze and assign a score to every study. Based on the number of RQs addressed, each study received a score accordingly, which formed the basis for the final quality assessment score. The score for every study ranges from 0 to 1, where 0 is the minimum score, while 1 is the maximum score a study can receive. The higher value of score increases the sincerity of the study. Each study scores one point for each research question addressed. Since we have seven research questions, a study can achieve seven points at maximum. Similarly, the quality assessment score of every study is based on (7) with mean according to the threshold in (8) for the final score. Hence, for addressing the research questions, a study can achieve a maximum score of 7 and a quality assessment score as 1.

The article "Taxonomy of Adaptive Neuro-Fuzzy Inference System in Modern Engineering Sciences" was retracted in 2023. Reasons: signs of a paper mill; compromised peer review; unreliable results or conclusions.

### 2.7. Data Synthesis

For the classification and arrangement of every piece of information from the selected studies related to our research questions, we employ data synthesis. We have primarily adopted two methods to synthesize our results:

- Narrative: we tabulate the results, after analyzing the data, incorporating various charts. RQ2, RQ3, RQ4, RQ5, and RQ6 belong to this category.
- Vote counting: we make some comparisons between the various models that are having higher research potential. RQ1 and RQ7 belong to this category.

### 2.8. Threat to Validity

#### 2.8.1. Study Selection Bias

Our defined search string is used in selecting the relevant studies for our SLR. We gave the best of our efforts in phrasing the search string in correspondence to our research questions. Yet, an existing possibility, where some relevant studies may have been missed, as per the fact that some studies had different keywords, in their title, abstract, and keywords, should be taken into account. Though we have emphasized avoiding such possibilities, using references from the bibliography of particular studies for the selection of all relevant studies, yet, there exists a probability that an important study may have been missed and as such is considered a threat.

#### 2.8.2. Subjective Quality Assessment

Quality assessment defines the criteria, by which we include and exclude the studies. This SLR also includes a possibility, in which several good quality studies might have been excluded. We try to minimize such threats, by scoring the studies based on our discussed criteria and making a final assessment based on the mean of those scores, thereby excluding only those studies, which fall below our set threshold criteria.

The article "Taxonomy of Adaptive Neuro-Fuzzy Inference System in Modern Engineering Sciences" was retracted in 2023. Reasons: signs of a paper mill; compromised peer review; unreliable results or conclusions.

## 3. Results and Discussions

The proposed research questions are discussed in this section.

### 3.1. What Are the Various ANFIS Hybrids? (RQ1)

The optimization algorithms are hybridized with existing techniques as a common practice. These techniques can be applied to various emerging domains. ANFIS can also be hybridized with such techniques proving its viability as a universal estimator.  Table 2 shows the summarized view of various ANFIS hybrids.

This table summarizes the various ANFIS hybrids, using optimization techniques, and their real-world applications. ANFIS widely adapts backpropagation for parameter optimization. Development of optimization algorithms revitalized the efforts to increase the accuracy of these systems, implicating that they can also address unique real-world problems, with human-like processing capability.

### 3.2. What Was the Purpose of Creating a Hybrid ANFIS Technique? (RQ2)

Real-world data is multidimensional, complex, and huge. The standard ANFIS uses Least Square Estimation and Gradient Descent to optimize its parameters, which can cause inaccurate prediction. This is due to the limitation that these algorithms converge slowly and compute time-consuming mathematical operations. To provide optimized solutions quickly in a large dataset, hybrid ANFIS techniques have been developed.

### 3.3. What Areas of Applications Have Been Touched by ANFIS Hybrids in the Real World? (RQ3)

ANFIS and its hybrids find widespread applications in several key areas of sciences and engineering.  Figure 3 demonstrates the share of applicability of ANFIS hybrids. From all the domains, Electronics has mostly embodied ANFIS followed by Geological Engineering. This suggests that ANFIS can be used to model complex real-world problems, e.g., software effort estimation [34] and intelligent systems.

### 3.4. What Are the Various Optimization Algorithm Hybrids of ANFIS? (RQ4)

Table 3 summarizes variants of the ANFIS hybrid techniques. The optimization techniques that extended the capabilities of ANFIS have been enhanced by hybridizing them with other optimization algorithms or various techniques to further improve their learning capability. ANFIS-PSO [28] has the most potential of advancing its capabilities because PSO [55] can be easily modified to include hybridized extensions. Hence, PSO can be combined with ANFIS when creating a variant, for accelerated computing ability. FFA [56] has also been favored by the researchers for extending capabilities of ANFIS.

The article "Taxonomy of Adaptive Neuro-Fuzzy Inference System in Modern Engineering Sciences" was retracted in 2023. Reasons: signs of a paper mill; compromised peer review; unreliable results or conclusions.

### 3.5. What Are the Possible Future Research Directions in context to ANFIS Current Literature Variants? (RQ5)

There are several hybrids of optimization techniques that are not yet implemented with ANFIS and are mentioned in Table 4. These algorithms are mostly hybridized variations of the standard optimization algorithms. PSO and BAT are widely hybridized and used to extend standard ANFIS architecture. ANFIS is a complementing framework for all technological paradigms and cross-cutting concerns. The exponential growth of data in recent years creates a thrust area to address issues of faster data processing capabilities, which can be handled well by ANFIS.

### 3.6. What Are the Current Trends in Research Based on ANFIS Techniques? (RQ6)

Figure 4 provides a trend of publications related to ANFIS techniques and its hybrids. The research remained stagnated for 14 years, up until 2007, when it was first combined with a hybrid of another popular technique, PSO, called Adaptive Weighted PSO. This suggests the viability of ANFIS in solving complex real-world problems as we move into automation and developing intelligent systems. The reason for the delayed usage of ANFIS in the scientific community is the presence of fewer data in the initial years of its invention. The research publication graph observes exponential growth as it delivers promising, effective, and accelerated results, a.k.a. solutions for various engineering and science domain optimization issues.

### 3.7. Which Hybrid Techniques Are the Most Popular in the Case of Implementations? (RQ7)

Figure 5 shows the count of ANFIS hybrids applied in different application areas. ANFIS-PSO has gained the highest popularity in the research community. The popularity of PSO has been exemplified here followed by ANFIS-ABC, ANFIS-FFA, and ANFIS-SC. The other hybrids as shown in Figure 5 are also successful trials.

## 4. Conclusion and Future Research Directions

ANFIS is one of the most promising algorithms to model human knowledge effectively, asserting its capabilities in complex problems that require manual intervention from humans. We have provided an exhaustive list of the most prominent ANFIS hybrids till date and their intended purpose by the authors. We further discussed the need to hybridize ANFIS, its usage in the current scenario and future scopes in modern engineering sciences. With the advent of metaheuristic optimization techniques, we discussed its advantages as compared to classical optimization methods and provided a comprehensive list of hybrids of these algorithms, which had been used further in ANFIS. The popularity of such metaheuristic techniques leads us to provide an analysis of the most sought-after algorithms that were used to hybridize ANFIS, with ANFIS-PSO and ANFIS-ABC as the topmost choices.

The article "Taxonomy of Adaptive Neuro-Fuzzy Inference System in Modern Engineering Sciences" was retracted in 2023. Reasons: signs of a paper mill; compromised peer review; unreliable results or conclusions.

We made an attempt to provide significant insights into the fields of implementations for ANFIS. It is assured that the future scope of research in ANFIS is having high potential. Electronics, Communication, and Geological fields of engineering have strived to adopt ANFIS, based on its amazing capabilities as a universal estimator. ANFIS can be opted for implementing Artificial General Intelligence; hence, its popularity is predicted to increase, as analyzed earlier in this paper.

## Figures and Tables

**Figure 1:** Methodology flowchart of the review protocol. This paper adheres to the steps mentioned in the figure, formulating a sequential presentation of the Systematic Literature Review (SLR). This methodology follows the standard process of reviewing literature and their selection for assuring quality review to the peers.

**Figure 2:** Standard structure of ANFIS. *w*1, *w*2, and *w*3 are the weights of the neurons and $\bar{w1}$, $\bar{w2}$, $\bar{w3}$ are the normalized weights of the neurons.

**Figure 3:** Share of application areas using ANFIS hybrids. This figure represents the average share of the various fields, where ANFIS has been implemented in real-world problems. ANFIS presents a wider potential for large scale, consumer-level product deployment, assisted by the advent in the field of Internet of Things (IoT) and 5^th^ Generation (5G) Networks.

**Figure 4:** History of publications on ANFIS (1993–2020). The wide research potential of the optimization algorithms led to an increase in publications in ANFIS.

**Figure 5:** Common implemented ANFIS hybrids. These selective hybrids are immensely implemented, in an attempt to develop solutions for several real-world problems.

**Table 1:** Advantages and disadvantages of ANFIS.

Advantages	Disadvantages
Captures nonlinearity of a process	Selecting type and number of membership functions
Automatic adaptation capability	Location of a membership function
Rapid learning capacity	Curse of dimensionality
High generalization capability	Interpretability-accuracy trade-off
High flexibility allows many variants	High computational cost

**Table 2:** Summary of prevailing ANFIS hybrids.

Model	Author	Abstract/findings
ANFIS	Roger Jang [2]	Automatic control system, adaptive signal processing, predictive coding, adaptive interference cancelling are few application areas of ANFIS
ANFIS-ABC (artificial bee colony)	Karaboga and Kaya [10]	It is used in updating the ANFIS parameter for the identification of nonlinear systems
ANFIS-ACO (ant colony optimization)	Cus et al. [11]	In the CNC machine process, determining the optimal machining parameters such as cutting speed, feed rate, and depth of cut
ANFIS-BA (BAT)	Premkumar and Manikandan [12]	It eliminates load variation issues and assists in speed control of brushless DC motor
ANFIS-BA (bees)	Marzia et al. [13]	Used in Mackey–Glass time-series prediction
ANFIS-BBO (biogeography-based optimization)	Ahmadlou et al. [14]	Providing the flood susceptibility maps in regions of Iran with high reasonable accuracies
ANFIS-CA (cultural algorithm) ANFIS-IWO (invasive weed optimization)	Khosravi et. al. [15]	In the Haraz watershed for identification of flood-prone areas with high precision
ANFIS-CBO (colliding bodies optimization)	Hassanzadeh et al. [16]	Used in estimating the bridge pier scour
ANFIS-COA (cuckoo optimization algorithm)	Mustapha [17]	Developing an algorithm for short-term electric load demand forecasting to improve forecasting accuracy and speed
ANFIS-CSA (crow search algorithm)	Elaziz et al. [18]	For any thermoacoustic heat exchanger in predicting the oscillatory heat transfer coefficient
ANFIS-CSA (cat search algorithm)	Orouskhani et al. [19]	Identification of nonlinear systems and prediction of a chaotic system
ANFIS-DE (differential evolution)	Zangeneh et al. [20]	Predicting Mackey–Glass time series and identification of a nonlinear dynamic system
ANFIS-FFA (firefly algorithm)	Yaseen et al. [21]	Assists in forecasting monthly rainfall with a one-month lead time
ANFIS-GA (genetic algorithm)	Hong et al. [22]	Development of an assessment for flood susceptibility, also using GIS with the technique
ANFIS-GWO (gray wolf optimization)	Jaafaria et al. [23]	For obtaining a reliable estimate of landslide susceptibility
ANFIS-HS (harmony search)	Wang et al. [24]	Epilepsy EEG signal classification
ANFIS-ICA (imperialist competitive algorithm)	Baseri and Belali-Owsia [25]	Predicting the output parameters of the manufacturing process
ANFIS-MFO (moth fly optimization)	Canayaz [26]	Solving problems of classification, nonlinear system identification, and time-series estimation
ANFIS-MHS (mosquito host seeking)	Sobia and Abudhahir [27]	Recognizing the facial expressions
ANFIS-PSO (particle swarm optimization)	Chen [28]	To construct a model for predicting business failures
ANFIS-SA (simulated annealing)	Haznedar and Kalinli [29]	Identifying dynamic systems
ANFIS-SBO (satin bowerbird optimizer)	Moosavi and Khatibi Bardsiri [30]	Software development effort estimation
ANFIS-SC (subtractive clustering)	Yadav and Ahmed [31]	Modeling academic performance in the educational domain
ANFIS-SFLA (shuffled frog-leaping algorithm)	Lin and Chen [32]	To build the MR damper inverse model
ANFIS-SSO (social spider optimization)	Ewees et al. [33]	To predict the biochar yield from manure pyrolysis

The article "Taxonomy of Adaptive Neuro-Fuzzy Inference System in Modern Engineering Sciences" was retracted in 2023. Reasons: signs of a paper mill; compromised peer review; unreliable results or conclusions.

**Table 3:** Optimization algorithm hybrids with their ANFIS counterparts.

Model	Variants
ANFIS-ABC [10]	ANFIS-aABC (adaptive ABC) [28, 29], ANFIS-Scoutless ABC [35]
ANFIS-ACO [11]	ANFIS-ACOr (ACO for continuous domains) [36, 37], ANFIS-ACS (ant colony system) [38]
ANFIS-BA [12]	HBA (hybrid bat algorithm)-ANFIS [39]
ANFIS-DE [20]	ANFIS-DEACS (differential evolution with ant colony search) [40]
ANFIS-FFA [21]	WT (wavelet transform)-ANFIS-HFPSO (hybrid FF and PSO) [41], MFA (modified FFA)-ANFIS-P&O (perturbation and observation) [42]
ANFIS-GA [22]	ANFIS-NSGAII (nondominated sorting GA-II) [35, 43]
ANFIS-HS [24]	ANFIS-GHS (global-best HS) [44]
ANFIS-PSO [28]	ANFIS-QPSO (quantum PSO) [45], ANFIS-QPSO-ADCEC (adaptive dynamical CE coefficient) [46], PSO-ANFIS-FFRLS (forgetting factor recursive least square) [47], ANFIS-adaptive weighted PSO [48], DyHAP (dynamic hybrid ANFIS-PSO) [49], wavelet-PSO-ANFIS [50], ANFIS-APAPSO (adaptive population activity PSO) [51]
ANFIS-SA [29]	ANFIS-RCSA (real-coded SA) [52]
ANFIS-SC [31]	TS (tabu search)-SC-ANFIS [53], ANFIS-FCM (fuzzy C-means) [54]

ANFIS, when hybridized with optimization algorithms, extends its error-handling capability, for accurate weight updating.

**Table 4:** Proposed hybrids of ANFIS implemented models.

Model	Model hybrids
ABC [57]	aABC [43, 58], adaptive ABC (AABC) [59], vortex search [60], cooperative ABC (CABC) [61, 62], cooperative micro-ABC (CMABC) [63], interval cooperative multiobjective ABC (ICMOABC) [62], ABC-PSO [64], multiobjective directed bee colony optimization (MODBCO) [65], Scoutless ABC [35], directed ABC [66, 67]
ACO [68]	ACOR [36], heuristic-PS-ACO (HPSACO) [69], hybrid ACO [70], ACO-PSO [71], PS-ACO [72], ACO-SA [73], MWIS-ACO-LS [74], hybrid ACO (HAntCO) [75], min-max ant System (MMAS) [72, 76], GA-ACO-SA [77], self-adaptive ant colony-genetic hybrid [78], GA-ACO [79], ACS [80], greedy ACS [81]
BA [82]	Binary BA [83], hybrid BA with ABC [84], BA-HS [85], adaptive BA [86], adaptive multiswarm BA (AMBA) [87], binary BA [83], differential operator & Levy flights BA [87], directed artificial BA (DABA) [88], double-subpopulation Levy flight BA (DLBA) [89], dynamic virtual BA (DVBA) [90], improved DVBA with probabilistic selection [91], island multipopulational parallel BA (IBA) [92], modified BA (stability analysis) [93], multiobjective BA (MOBA) [94], novel BA with multiple strategies coupling (mixBA) [95], OBMLBA [96], shrink factor BA (SBA) [92], simplified adaptive BA based on frequency [97]
DE [98]	DE with modified PSO (DEMPSO) [99], DEPSO [100], DE-GA [101], DE with K-means clustering [102], DE-GWO [103], DE with adaptive mutation (DEAM) [104], simplified real-coded differential GA (SADE) [105], DEACS [40]
FFA [56]	Hybrid firefly with PSO (HFPSO) [106], modified FFO (MFO) [107], FA-HS [108]
GA [109]	HGA with local search [110], adaptive HGA (a-HGA) [111], GSA-GA [112], GA/SA [113], GA/SA/TS [114], GA-PSO [115]
HS [116]	GHS [117], HS-teaching-learning-based optimization (HSTLBO) [118], HS-SA [119], mutation-based HS (MBHS) [120], GWO-HS [121], hybrid Taguchi-HS [122], HS-BA [85]
PSO [55]	APAPSO [51], PSO-LMS [123], QPSO [124], IQPSO [125], PSO-SA [126], PSO-BFO [123], GA-PSO [127], PSO-FLC [128], enhanced PSO [127], DEMPSO [99], DEPSO [100], PSO-local search [129]
SA [130]	Integer augmented SA (IASA) [131], real-coded augmented SA (RASA) [131], real-coded SA (RCSA) [52]
SC [132]	SC-FCM (subtractive clustering-fuzzy C-means) [133], FCM-ELPSO [134], firefly-based FCM (FFCM) [135]

Optimization algorithms form the backbone of Artificial Neural Networks (ANNs). They help correctly update the weights of the network neurons, so that the prediction improves. Backpropagation is a widely popular and simple optimization algorithm. It is utilized heavily in popular Deep Learning frameworks PyTorch and TensorFlow. Limitations of backpropagation provided the research community to develop several alternatives, such as ACO, PSO, GA, and BAT.

The article "Taxonomy of Adaptive Neuro-Fuzzy Inference System in Modern Engineering Sciences" was retracted in 2023. Reasons: signs of a paper mill; compromised peer review; unreliable results or conclusions.

## Data Availability

The data shall be made available upon request.
